The article "Impact of varying levels of soil salinity on emergence, growth and biochemical attributes of four Moringa oleifera landraces" was retracted in 2022. Reasons: compromised peer review; a conflict of interest; concerns about the authorship.

# Impact of varying levels of soil salinity on emergence, growth and biochemical attributes of four *Moringa oleifera* landraces

**DOI:** 10.1371/journal.pone.0263978

**Published:** 2022-02-22

**Authors:** Fatima Farooq, Nabila Rashid, Danish Ibrar, Zuhair Hasnain, Rehmat Ullah, Muhammad Nawaz, Sohail Irshad, Shahzad M. A. Basra, Mona S. Alwahibi, Mohamed S. Elshikh, Helena Dvorackova, Jan Dvoracek, Shahbaz Khan

**Affiliations:** 1 Department of Botany, University of Agriculture, Faisalabad, Pakistan; 2 National Agricultural Research Centre, Islamabad, Pakistan; 3 Department of Agronomy, PMA-Shah Arid Agriculture University, Rawalpindi, Pakistan; 4 Soil and Water Testing Laboratory for Research, Dera Ghazi Khan, Pakistan; 5 Department of Agricultural Engineering, Khwaja Fareed University of Engineering and Information Technology, Rahim Yar Khan, Pakistan; 6 Department of Agronomy, MNS-University of Agriculture, Multan, Pakistan; 7 Department of Agronomy, University of Agriculture, Faisalabad, Pakistan; 8 Department of Botany and Microbiology, College of Science, King Saud University, Riyadh, Saudi Arabia; 9 Department of Agrochemistry, Soil Science, Microbiology and Plant Nutrition, Faculty of AgriSciences, Mendel University in Brno, Brno, Czech Republic; 10 Pedologiejh, spol s.r.o, Brno, Czech Republic; Anhui Agricultural University, CHINA

## Abstract

Salinity in soil and water is one of the environmental factors that severely hinder the crop growth and production particularly in arid and semi-arid regions. A pot experiment was conducted to investigate the impact of salinity levels (1.5 dS m^-1^, 3.5 dS m^-1^, 7.5 dS m^-1^ and 11.5 dS m^-1^) on emergence, growth and biochemical traits of moringa landraces under completely randomized design having three replications. Four landraces of *Moringa oleifera* (Faisalabad black seeded moringa [MFB], Patoki black seeded moringa [MPB], Faisalabad white seeded moringa [MFW] and Rahim Yar Khan black seeded moringa [MRB]) were selected for experimentation. All the salinity levels significantly affected the emergence parameters (time to emergence start, time to 50% emergence, mean emergence time, emergence index and final emergence percentage) of moringa landraces. However, 1.5 dS m^-1^ and 3.5 dS m^-1^ were found more favorable. Higher salinity levels (7.5 dS m^-1^ and 11.5 dS m^-1^) significantly minimized the root surface area, root projected area, root volume and root density as compared to 1.5 dS m^-1^, 3.5 dS m^-1^. Number of branches, leaves, leaflets and leaf length were also adversely affected by 7.5 dS m^-1^ and 11.5 dS m^-1^. Maximum seedling fresh and dry weights, and seedling length were recorded at 1.5 dS m^-1^ followed by 3.5 dS m^-1^. Chlorophyll *a* and *b* contents, carotenoids and membrane stability index were also observed highest at salinity level of 1.5 dS m^-1^. In case of moringa landraces, MRB performed better regarding emergence attributes, growth parameters, and biochemical analysis followed by MFW as compared to MFB and MPB. Moringa landraces i.e. MRB and MFW were found more tolerant to salinity stress as compared to MFB and MPB.

The article "Impact of varying levels of soil salinity on emergence, growth and biochemical attributes of four Moringa oleifera landraces" was retracted in 2022. Reasons: compromised peer review; a conflict of interest; concerns about the authorship.

## Introduction

Urbanization is a major threat for agriculture sustainability because agricultural land is being ruthlessly used for commercial purposes [1]. At the same time, various abiotic stresses like soil salinity, drought, extreme temperature and high wind are adversely influencing the production and cultivation of field crops. Among these, salinity is one of the most destructive environmental stress, which causes the reduction of crop yield and its quality [1]. Salinization is considered as a major abiotic stress, especially in semi-arid and arid regions, that affects plant growth throughout the world [2, 3]. Salt stress affects the water uptake, decreases photosynthetic rate and synthesis of photosynthetic pigments resulting in reduction of plant growth [4]. It also reduces the stomatal conductance, thereby limiting CO_2_ supply to leaves as well inhibits PSII activities [5]. Salinity leads to cause osmotic stress and ionic toxicity which adversely affects growth and economic yield of plants [6]. In Pakistan, salinity stress is at an alarming rate because total cultivated area is 22.1 Mha out of which 6.28 Mha area is salt affected [7]. Human activities are also responsible for secondary salinization by mishandling the land and primary source of salinity [8]. As salt concentration increases in soil, uptake of Zn is decreased and Cd toxicity increases in plants which have deleterious effects on plant growth and development [9].

*Moringa oleifera* is a perennial tree, commonly known as horseradish found in tropical and sub-tropical regions. It is source of herbal medicine because it is rich in antioxidant like ascorbic acid, tocopherols (Vitamin E) and minerals, and also used as vegetable [10]. There are several clinical studies on moringa trees focused on its pharmacological role in osteoporosis, anemia and diabetes mellitus. Moringa leaves have different therapeutic applications such as antiparasitic, anti-oxidant, anti-inflammatory, antibacterial, antifungal and cardioprotective activities [11]. Moringa leaf extract and root extract are also being used as crop growth enhancer either through foliar application and /or seed priming agents to improve the growth and productivity of field crops [12–15]. Moringa plant may resistant to moderate saline condition [16] but when it is exposed to high salt concentration it behaves as a salt sensitive crop [17]. Under high salinity, uptake of K^+^ and Ca^2+^ is restricted in moringa plants with low dry weight, less root and shoot length [18]. In some moringa landraces, photosynthetic pigments also affected under high salinity [19].

The article "Impact of varying levels of soil salinity on emergence, growth and biochemical attributes of four Moringa oleifera landraces" was retracted in 2022. Reasons: compromised peer review; a conflict of interest; concerns about the authorship.

To overcome the impact of salinity, various agronomic and genetic approaches are being practiced worldwide [20–22]. Among those, one of them is cultivation of salt resistant flora. According to our best knowledge there is no study about salinity tolerance of different moringa landraces at various salinity levels. This study was planned to explore the impact of various levels of salt stress on growth and development of different moringa landraces present in Pakistan. The present study also investigated the growth and physiological response of different moringa landraces in saline conditions and to determine the optimum, lethal and sub-lethal levels of salt stress.

## Materials and methods

### Experimental particulars

Experiment was conducted in the wire house, Department of Agronomy, University of Agriculture, Faisalabad to evaluate the adverse effect of sodium chloride on different landraces of moringa. Four landraces of *Moringa oleifera* (Faisalabad black seeded moringa [MFB], Patoki black seeded moringa [MPB], Faisalabad white seeded moringa [MFW] and Rahim Yar Khan black seeded moringa [MRB]) were selected for experimentation and their seeds were collected from their respective places. Completely randomized design (CRD) with three replications was followed to conduct the experimentation. Four salinity levels i.e. 1.5 dS m^-1^, 3.5 dS m^-1^, 7.5 dS m^-1^ and 11.5 dS m^-1^ were under study. Salinity level of 1.5 dS m^-1^ was considered as control. Fifteen seeds of each landrace were sown in the pots having 5 kg of soil on March 8, 2019. The plants were grown for a period of one month under natural conditions in wire house. During this period of growth each pot was irrigated by 150 ml of water daily. Four salinity levels (1.5 ds m^-1^, 3.5 dS m^-1^, 7.5 dS m^-1^ and 11.5 dS m^-1^) were created by adding calculated amount of NaCl salt and mixing manually according to procedure mentioned in USDA laboratory manual [23]. Three plants from each replication were randomly selected to record the data regarding seedling emergence, growth, physiological attributes and biochemical analyses.

### Emergence parameter

Daily emerged seeds were counted until the final seed emerged and following parameters were recorded. Emergence was counted on daily basis until a constant count achieved. Time to start emergence and time taken for 50% germination (T50) were measured according to Farooq *et al*. [24] formula; [T50 = ti + {(N/2 − ni)/ (nj − ni)} × (tj − ti)]. Mean emergence time (MET) was calculated [25] (MGT = Dn/n). Emergence index (EI) was calculated by AOSA [26] [EI = (number of germinated seed(s)/day of first count) + …. + (number of germinated seeds/days of final count)]. Final emergence percentage was calculated according to formula (FEP = Final no. of seeds germinated / total number of seeds) [27].

The article "Impact of varying levels of soil salinity on emergence, growth and biochemical attributes of four Moringa oleifera landraces" was retracted in 2022. Reasons: compromised peer review; a conflict of interest; concerns about the authorship.

### Growth, physiological and biochemical analysis

Randomly selected three plants from each pot were observed for their physiological and biochemical analysis. The growth attributes were recorded after one month of emergence. Seedlings fresh weight was recorded at the time of harvesting and dry weight was measured by oven drying the samples until the constant weight obtained. Growth parameters like root length, plant height, leaflet length, number of leaves per plant, number of leaflets per leaf, number of branches per plant were recorded at harvesting stage. Root length, surface area, projected area, average density and volume were measured by using root scanner (STD4800). To determine the chlorophyll *a* and *b* and carotenoids, the leaves were taken from each replication and kept in freezer overnight for chilling rupture. The 0.1 g sample form these leaves was taken and dipped in 5 ml of 80% acetone solution and centrifuged for 15 minutes at 10,000 x g. After that, the data were recorded using the UV-visible spectrophotometer against a blank containing 80% acetone at wavelength 480, 645 and 663 nm [28].

### Statistical analysis

Collected data regarding emergence, growth, physiological and biochemical attributes were analyzed and evaluated statistically by using statistical package “Statistic 8.1” by employing the Fisher’s analysis of variance (ANOVA) technique at 5% probability level under completely randomized design [29]. Treatments’ means were compared using Tukey Honest Significant Difference (HSD). Microsoft Excel was used for calculation and graphical presentation.

## Results

In present study, effect of four salinity levels (1.5, 3.5, 7.5 and 11.5 dS m^-1^) were observed on emergence and seedling vigor of four moringa landraces (MFB, MPB, MFW and MRB). The significance of salinity levels and moringa landraces as well as their interaction is presented in Table 1. It has been observed that salinity levels significantly affected the emergence parameters (time to emergence start, time to 50% emergence, mean emergence time, emergence index and final emergence percentage) of all moringa landraces at various extent. Overall, at highest salinity level (11.5 dS m^-1^), moringa seeds took maximum time for emergence than at control (lowest salinity level; 1.5 dSm^-1^). Similarly, emergence index (EI) and final emergence percentage (FEP) were also recorded best at lowest salinity level as compared to highest salinity level. Moreover, all moringa landraces showed different emergence rate at different salinity level, thus maximum emergence attributes were recorded in MFB followed by MPB, MFW and MRB (Fig 1).

The article "Impact of varying levels of soil salinity on emergence, growth and biochemical attributes of four Moringa oleifera landraces" was retracted in 2022. Reasons: compromised peer review; a conflict of interest; concerns about the authorship.

**Fig 1:** Impact of salinity on time to start emergence (TSE), time to 50% emergence time (T50), mean emergence time (MET), emergence index and final emergence percentage (FEP) of moringa landraces.

**Table 1:** Mean sum of squares of emergence, growth and physiological parameters of moringa landraces grown under varying salinity levels.

SOV	DF	TSE	T50	MET	EI	FEP	RSA	RPA	RV	RD	NB
Salinity levels (SL)	3	100.13**	21.25**	36.31**	24.07**	1211.39**	703.12**	69.89**	0.077**	0.16**	46.46**
Landraces (LR)	3	8.47**	35.06**	88.36**	5.24**	49.28**	137.87**	12.81**	0.022**	0.013**	3.62**
SL × LR	9	2.28^NS^	0.47^NS^	1.50^NS^	0.21^NS^	6.26^NS^	232.25**	3.17**	0.012**	0.0042**	0.403^NS^
		NL	NLL	LL	SFW	SDW	SL	Chl *a*	Chl *b*	CAR	MSI
Salinity levels (SL)	3	54.83**	72.35**	29.83**	2782.06^NS^	315.970**	4242.06**	6.97^NS^	0.0829**	1.55021	1855.10**
Landraces (LR)	3	3.94**	5.41**	0.716**	7.75**	5.388**	84.71**	0.0057**	0.034**	0.0096 ^NS^	18.35**
SL × LR	9	0.33^NS^	1.15^NS^	0.329*	11.88^NS^	0.633^NS^	16.42^NS^	0.060**	0.0187**	0.0094*	3.02**

SOV = Source of variance, DF = Degree of freedom, Chl = Chlorophyll, CAR = Carotenoids, TSE = Time to start emergence, T50 = 50% emergence time, MET = Mean emergence time, EI = Emergence index, FEP = Final emergence percentage, RSA = Root surface area, RPA = Root projected area, RV = Root volume, RD = Root density, NL = No of leaves per plant, NB = No of branches, NLL = no of leaflets per plant, LL = leaf length, SFW = Seedling fresh weight, SDW = Seedling dry weight, SL = Seedling length, MSI = Membrane stability index, NS = Non-significant

* = Significant at P ≤ 0.05

** = Significant at P ≤ 0.01.

The effect of various salinity levels (1.5, 3.5, 7.5 and 11.5 dSm^-1^) was observed on morphological attributes of moringa landraces (MFB, MPB, MFW, MRB). Data recorded for seedling fresh weight demonstrated that all moringa landraces showed maximum fresh biomass at minimum salinity level (1.5 dS m^-1^), while least seedling fresh weight was observed at highest salinity level (11.5 dS m^-1^). Similarly, the results obtained for seedling dry weight was showed that among different moringa landraces maximum seedling dry weight was noted at 1.5 dS m^-1^ salinity level, while least was observed at 11.5 dS m^-1^ salinity level. However, the order of improvement of seedling dry weight among landraces was: MBR > MPB > MFW > MFB. Data, recorded for seedling length, showed significant difference between moringa landraces and salinity levels but their interaction was non-significant. Among the salinity levels the plant showed the maximum seedling length at minimum salinity level (1.5 dS m^-1^), while the maximum seedling length of MBR landrace was noted as compared to other landraces. However, at highest salinity level (11.5 dS m^-1^) maximum reduction in seedling length was recorded (Fig 2).

The article "Impact of varying levels of soil salinity on emergence, growth and biochemical attributes of four Moringa oleifera landraces" was retracted in 2022. Reasons: compromised peer review; a conflict of interest; concerns about the authorship.

**Fig 2:** Impact of salinity on time to seedling fresh weight, seedling dry weight and seedling length of moringa landraces.

Data, recorded for chlorophyll contents, showed that salinity levels decreased the chlorophyll *a* content of all landraces. All the landraces showed different behavior under salinity levels, the order reduction among all moringa landraces at 1.5 dS m^-1^ salinity level was: MPB > MFB > MRB > MFW, while order of reduction at 3.5 dS m^-1^ was: MFB > MBP > MFW > MRB, at 7.5 dS m^-1^ salinity level reduction order was: MRB > MFB > MFW > MPB, similar at 11.5 dS m^-1^ salinity level reduction order was: MFW > MRB > MPB > MFB. Thus overall, maximum chlorophyll *a* content was noted in MFW landrace and MPB synthesized minimum chlorophyll *a* pigment. Moreover, data recorded for chlorophyll *b* showed that among all moringa landraces, maximum chlorophyll *b* pigments were observed in MFW while MBP had minimum chlorophyll *b* contents. Results obtained for carotenoids concentration showed that among moringa landraces, MRB showed maximum carotenoids while MFW showed minimum. However highest carotenoids concentration was noted at 7.5 dS m^-1^ salinity level and lowest concentration was observed at 11.5 dS m^-1^ salinity level. Membrane stability index (MSI) was significantly different among the salinity level, lowest reduction of MSI noted at 3.5 dS m^-1^ salinity level and highest reduction was observed at 11.5 dS m^-1^. Among all moringa landraces, MRB showed more MSI, while MPB had least MSI value (Fig 3).

**Fig 3:** Impact of salinity on chlorophyll *a* and *b* contents, carotenoids and membrane stability index of moringa landraces.

Data showed that higher soil salinity significantly decreased the root surface area (RSA) of all moringa landraces. Among all salinity level maximum RSA was observed at 1.5 dS m^-1^ salinity level, while minimum RSA was noted at highest salinity level i.e. 11.5 dS m^-1^. However, among all moringa landraces the order of RSA was: MRB > MFB > MFW > MPB. Data noted for root projected area (RPA) showed significant difference among salinity levels and moringa landraces. Maximum reduction in RPA was observed at 11.5 dS m^-1^. Maximum RPA was observed in MRB landrace followed by MFB, MFW and MPB. Results obtained for root volume (RV) demonstrated that there was significant difference between salinity levels as well as moringa landraces. Salinity levels significantly decreased the RV of all moringa landraces, but highest reduction was noted at 11.5 dS m^-1^ salinity level. Moreover, maximum RV was observed in MRB landrace followed by MPB, MFW and MFB landraces. Similarly, salinity levels significantly affect the root density (RD) of moringa landraces, maximum reduction was observed in MFW landrace at 11.5 dS m^-1^ salinity level, while highest RD was noted in MFB landrace at minimum salinity level i.e. 1.5 dS m^-1^ (Table 2). Salinity significantly decreased the total number of branches, leaves, leaflets and leaf length of all moringa landraces, but maximum reduction was recorded at 11.5 dS m^-1^ salinity level and least reduction was observed at 1.5 dS m^-1^ salinity level. There was also significant difference among the landraces. Highest number of branches, leaves and leaf length was noted in MRB moringa, while maximum number of leaflets was observed in MFW moringa landrace (Table 3).

The article "Impact of varying levels of soil salinity on emergence, growth and biochemical attributes of four Moringa oleifera landraces" was retracted in 2022. Reasons: compromised peer review; a conflict of interest; concerns about the authorship.

**Table 2:** Impact of various salinity levels on root attributes of moringa landraces.

**Treatments**	**Root surface area (cm** ^**2**^ **)**					**Root projected area (cm** ^**2**^ **)**				
	MFB	MPB	MFW	MRB	Mean (SL)	MFB	MPB	MFW	MRB	Mean (SL)
1.5 d Sm^-1^	26.36a	13.99de	23.23ab	21.69bc	21.19A	7.05a	3.67d-f	4.06c-e	7.9633a	5.69A
3.5 d Sm^-1^	16.69de	6.92f	13.00e	17.73cd	13.58C	6.59ab	4.58b-d	6.41ab	5.88a-c	5.86A
7.5 d Sm^-1^	7.32f	5.48fg	5.65fg	13.99de	8.11C	2.28e-g	1.58fg	1.39g	4.43b-e	2.42 B
11.5 d Sm^-1^	3.99fg	1.91g	2.82g	4.78fg	3.37D	1.18g	0.812g	0.67g	1.405g	1.02C
Mean (LR)	13.591 A	6.949 C	11.174 B	14.548 A		4.27A	2.6632 B	3.1337 B	4.92A	
HSD	SL = 1.6128, LR = 1.4506, SL×LR = 3.9738					SL = 0.5387, LR = 0.8057, SL×LR = 2.2071				
**Treatments**	**Root volume (cm** ^**3**^ **)**					**Root density**				
	MFB	MPB	MFW	MRB	Mean (SL)	MFB	MPB	MFW	MRB	Mean (SL)
1.5 d Sm^-1^	0.15de	0.29a	0.28a-c	0.33a	0.2567 A	0.5127 a	0.4660 b	0.4550 b	0.4427 b	0.4691 A
3.5 d Sm^-1^	0.102d-g	0.26ab	0.135d-f	0.27a	0.1931 B	0.5377 a	0.3967 c	0.3697 c	0.4453 b	0.4373 B
7.5 d Sm^-1^	0.17b-d	0.09d-g	0.039g	0.17cd	0.1193 C	0.4590 b	0.3743 c	0.3987 c	0.4613 b	0.4233 B
11.5 d Sm^-1^	0.09d-g	0.06fg	0.66e-g	0.09d-g	0.0753 D	0.2050 d	0.2057 d	0.2187 d	0.2187 d	0.2123 C
Mean (LR)	0.1280 C	0.1769 B	0.1246 C	0.2149 A		0.4286 A	0.3607 C	0.3605 C	0.3922 B	
HSD	SL = 0.0417, LR = 0.0322, SL×LR = 0.0883					SL = 0.0218, LR = 0.0149, SL×LR = 0.0408				

The article "Impact of varying levels of soil salinity on emergence, growth and biochemical attributes of four Moringa oleifera landraces" was retracted in 2022. Reasons: compromised peer review; a conflict of interest; concerns about the authorship.

**Table 3:** Impact of various salinity levels on growth attributes of moringa landraces.

**Treatments**	**Number of branches**					**Number of leaves**				
	MFB	MPB	MFW	MRB	Mean (SL)	MFB	MPB	MFW	MRB	Mean (SL)
1.5 d Sm^-1^	7.67	7.00	6.67	8.67	7.5A	8.33	7.67	8.33	9.67	8.50 A
3.5 d Sm^-1^	7.00	6.33	7.00	7.67	7.0A	7.0	7.33	7.00	8.33	7.42 B
7.5 d Sm^-1^	4.67	3.67	4.17	5.33	4.46A	5.0	4.67	4.00	5.33	4.75 C
11.5 d Sm^-1^	3.33	3.33	3.33	3.67	3.42C	4.0	3.67	3.67	4.67	4.00 C
Mean (LR)	5.67 AB	5.08 B	5.29 B	6.33 A		6.08 B	5.83 B	5.75 B	7.00 A	
HSD	SL = 1.0174, LR = 1.0239, SL×LR = 2.8048					SL = 0.7603, LR = 0.8904, SL×LR = 2.4391				
**Treatments**	**Number of leaflets**					**Leaf length**				
	MFB	MPB	MFW	MRB	Mean (SL)	MFB	MPB	MFW	MRB	Mean (SL)
1.5 d Sm^-1^	10.0	9.66	11.33	10.0	10.25A	8.33ab	7.67a-c	8.3333 ab	9.67a	8.5A
3.5 d Sm^-1^	7.0	7.667	10.0	9.33	8.5B	7.0b-e	7.33a-d	7.0b-e	8.33ab	7.42B
7.5 d Sm^-1^	5.33	5.667	5.67	6.0	5.67C	5.0d-f	4.66ef	4.0f	5.33c-f	4.75C
11.5 d Sm^-1^	4.33	4.667	5.33	5.67	5.0C	4.0f	3.66f	3.67f	4.66ef	4.0C
Mean (LR)	6.66B	6.92B	8.08A	7.75AB		6.08B	5.83B	5.75B	7.0A	
HSD	SL = 1.0617, LR = 1.0854, SL×LR = 2.9733					SL = 0.3841, LR = 0.4178, SL×LR = 1.1446				

## Discussion

Salinity is also known to impair seed germination, emergence and early seedling growth [30]. The presence of more salt in the soil negatively affected physiological and biochemical attributes in plants which decreased plant biomass and economic yield [31]. Various plants have different salt tolerance levels, as do most cereals, including moringa. The results of present study depict that, the speed and spread of seedling of different moringa landraces were reduced with increasing salinity (Fig 1). These results corroborate the findings of previous studies that higher salt stress retards seed germination and seedling emergence rate, emergence index due to osmotic effect, which is deleterious and prevents the plant in maintaining their proper nutritional requirements necessary for seedling vigor [32, 33]. Salt stress delayed the seedling germination, lower seedling growth rate resulting in hampered crop growth and yield, because salinity lowered the soil water potential [34, 35] as well as increase Na^+^ level in plant cells which limit plant productivity, in severe plant death occur [36].

A stronger root system could probably lead to more plant biomass production on normal growth conditions or less yield reduction under abiotic stress and nutrient-deficient conditions. Root development requires uptake, translocation, and metabolism of essential nutrients. The development of root system architecture is a biological process that interacts with ion homeostasis [37]. In this study, root surface area, root projected area, root volume and density significantly affected by increasing the salinity concentration in soil in all moringa landraces (Fig 2). Minimum root attributes were affected in MRB moringa landrace, this may be due to genetically strong adaptation as compared to other landraces, while root length was severely affected by salt stress. Similarly, salt stress affected the root architecture in wheat cultivars due to ionic imbalance [37]. Moreover, it has been found that salinity reduced the root density and root surface area [38] and root density [39, 40] in plants. It is also reported that organic amendments play a vital role to reduce the impact of abiotic stress [41, 42].

The article "Impact of varying levels of soil salinity on emergence, growth and biochemical attributes of four Moringa oleifera landraces" was retracted in 2022. Reasons: compromised peer review; a conflict of interest; concerns about the authorship.

Generally, salinity is known to cause a marked reduction in photosynthetic (chlorophyll *a*, *b*) and accessory pigments (carotenoids) as noted in present study (Fig 3). High salt concentration caused the formation of chlorophyllase and hampered nitrogen absorption which disturb the biosynthesis of photosynthetic pigments which adversely affect photosynthetic rate and ultimately limited crop yield [43, 44]. Salt stress changed the ultrastructure of cellular components by enhancing the reactive oxygen species (ROS) which cause lipid peroxidation of plasma membrane, ultimately photosynthetic machinery disturbed, resulting growth and economic yield of plants reduced [45]. At high salinity levels, crude protein, carotenoids and chlorophyll were reduced while antioxidants, enzymes, non-enzymes, proline and total carbohydrates were also increased [19]. Sustainable production is possible if integrated application of agronomic and cultural practices is insured [46].

The general effect of salinity is to reduce the growth rate resulting in smaller leaves, shorter stature, and sometimes fewer leaves. Moringa plants may resistant to moderate saline condition [16] but when it is expose to high salt concentration its growth decreased [17] which was in line with results of current study in which salinity stress effects the growth and development of moringa landraces. Because high salinity level inhibits the uptake of K^+^ and Ca^2+^ as well as enhance Na^+^ toxicity, which hamper plant crucial mechanism [47], as a consequence plant length and fresh and dry biomass affected [18]. Plant growth decreased by increasing the level of salinity, all landraces showed lower seedling length and fresh dry biomass. It is also reported that unfavorable conditions significantly reduced the emergence and growth attributes [48].

Nevertheless, MRB landrace had improved seedling growth compared to other landraces. The reduction in plant length, fresh and dry weight may be due to increase of Na^+^ ion toxicity, loss of cell membrane permeability and senescence [49–51]. Environmental stress is responsible for reduction in the growth and development of crops [52]. It has been reported that Na^+^ toxicity significantly hampered the photosynthesis process, resulting in energy supply to plant body reduced, hence shoot and root growth decreased [36]. The results of the present study show that the growth of moringa landraces (number of branches, leaves, leaflets and leaf length) was decreased significantly with increasing salinity levels in all landraces, resulting limited plant growth. Overall, MRB showed better adaptation as compared to other landraces. Similar findings were also reported on various plants which were in line with our results [53, 54].

The article "Impact of varying levels of soil salinity on emergence, growth and biochemical attributes of four Moringa oleifera landraces" was retracted in 2022. Reasons: compromised peer review; a conflict of interest; concerns about the authorship.

## Conclusion

In present study, impact of four salinity levels (1.5, 3.5, 7.5 and 11.5 dS m^-1^) were observed on seedling emergence, growth and biochemical attributes of four landraces of *Moringa oleifera* (Faisalabad black seeded moringa [MFB], Patoki black seeded moringa [MPB], Faisalabad white seeded moringa [MFW] and Rahim Yar Khan black seeded moringa [MRB]). It can be concluded from the results of current experimentation that moringa can tolerate the salinity up to 3.5 dS m^-1^ and retain optimum growth. Its growth is adversely affected as the salinity level increases up to 7.5 dS m^-1^. Regarding moringa landraces, Rahim Yar Khan black seeded moringa and Faisalabad white seeded moringa are more resistant to salinity stress as compare to Faisalabad black seeded moringa and Patoki black seeded moringa.
